The article "Bufalin, a component in Chansu, inhibits proliferation and invasion of hepatocellular carcinoma cells" was published in 2013. Journal: BMC Complement Altern Med.

# Bufalin, a component in Chansu, inhibits proliferation and invasion of hepatocellular carcinoma cells

**DOI:** 10.1186/1472-6882-13-185

**Published:** 2013-07-19

**Authors:** Dong-Ze Qiu, Zhou-Ji Zhang, Wei-Zhong Wu, Yun-Ke Yang

**Affiliations:** 1 Department of Traditional Chinese Medicine, Zhongshan Hospital, Fudan University, Shanghai 200032, PR China; 2 Key Laboratory of Carcinogenesis and Cancer Invasion, Ministry of Education, Liver Cancer Institute and Zhongshan Hospital, Fudan University, Shanghai 200032, PR China

**Keywords:** Hepatocellular carcinoma, Bufalin, Proliferation, Invasion, AKT signaling pathway

## Abstract

**Background:**

Hepatocellular carcinoma (HCC) is a common and aggressive cancer, and the treatment options are limited for patients with advanced HCC. Bufalin, the major digoxin-like component of the traditional Chinese medicine Chansu, exhibits significant anti-tumor activities in many tumor cell lines. In the present study, we investigated the effect of bufalin on the inhibition of an AKT-related signaling pathway, and examined the relationship between regulatory proteins and anti-tumor effects in hepatoma cells.

**Methods:**

Proliferation, wound healing, transwell-migration/invasion and adhesion assays were performed in HCCLM3 and HepG2 cell lines. The protein levels of pAKT, AKT, pGSK3β, GSK3β, pβ-catenin, β-catenin, E-cadherin, MMP-9, and MMP-2 were measured by western blot analysis. E-Cadherin and β-catenin expression levels were also evaluated by immunofluorescence.

**Results:**

Bufalin inhibited hepatoma cell proliferation, migration, invasion and adhesion. In addition, treatment with bufalin significantly decreased the levels of pAKT, pGSK3β, MMP-9, and MMP-2, while increasing the levels of GSK3β and E-cadherin and suppressing the nuclear translocation of β-catenin.

**Conclusions:**

Bufalin is a potential anti-HCC therapeutic candidate through its inhibition of the AKT/GSK3β/β-catenin/E-cadherin signaling pathway. Further studies with bufalin are warranted in patients with HCC, especially those with the disease at advanced stages.

## Background

Hepatocellular carcinoma (HCC) is one of the main causes of cancer mortality in many countries, especially in East and Southeast Asia and Central and West Africa [1]. HCC is the fifth most common cancer in men and the seventh most common in women, and is the third leading cause of cancer death [2]. The disease is usually diagnosed at an advanced stage and recurrence rates are very high; approximately 30–40% within 5 years. Patients with advanced HCC have a median survival of about 6–8 months, and there are limited effects in the treatment for these patients [3]. 5-Fluorouracil and mitomycin-C, widely used chemotherapeutic drugs, have limited overall effects in the treatment of HCC owing to resistance. Nowadays, patients with advanced HCC are treated with a comprehensive series of vascular interventional therapy, but their median life spans are not obviously prolonged [4]. Certain Chinese traditional medicines were found to be effective in treatment on cancers, drugs like Songyou Yin which were reported to improve the efficacy of chemotherapy in HCC [5]. Therefore, novel therapeutic strategies are essential to improve the clinical management of patients with HCC.

Bufalin, the major digoxin-like component of the traditional Chinese medicine Chansu, is an extract from the skin and parotid venom glands of *Bufo bufo gargarizans cantor*[6]. Chansu, initially recorded more than 1000 years ago, is a well-known traditional Chinese medicine widely used in clinical cancer therapy in China [7,8]. Recent experimental studies have suggested that Chansu and its active compounds exhibit significant anti-tumor activity via the inhibition of cell proliferation, induction of cell differentiation and apoptosis, disruption of the cell cycle, inhibition of angiogenesis, reversal of multidrug resistance, and regulation of the immune response [9]. In a previous study, it was demonstrated that bufalin caused apoptosis of gastric cancer cells by inhibition of the AKT signaling pathway via CBL-B and CBL-C [10]. AKT (also known as PKB) is a master regulator that when activated by phosphorylation modifies at least 10 major regulatory proteins and initiates many pathways in tumor cells [11]. PI3K/AKT signaling is involved in the regulation of cancer cell proliferation, motility, survival and metabolism [12,13]. AKT is also instrumental in angiogenesis and epithelial mesenchymal transitions during tumorigenesis [13,14].

The purpose of this study was to observe the anti-tumor effects and molecular mechanisms of bufalin in hepatoma cells, especially the AKT signaling pathway.

## Methods

### Cell lines

The human hepatoma cell lines HCCLM3 and HepG2 were provided by the Liver Cancer Institution, Zhongshan Hospital, Fudan University (Shanghai, China) and were used in all experiments. Both cell lines were cultured in Dulbecco’s modified Eagle’s medium (DMEM) supplemented with 10% fetal bovine serum (FBS) at 37°C in a humidified atmosphere of 5% CO_2_ and 95% air.

### Compounds and antibodies

Bufalin (purity >98%) was purchased from Shanghai Tauto Biotech Co., Ltd. (Shanghai, China), dissolved in ethanol at a concentration of 10^–2^ mol/L, sterilized with a 0.22-μm filter (Millipore, Billerica, MA, USA), and stored at 4°C. Figure 1 shows the chemical structure of bufalin. Antibodies against GSK3β, pGSK3β (Ser 9), β-catenin, pβ-catenin (Ser 33/37), GAPDH, and E-cadherin were purchased from Epitomics Inc. (Burlingame, CA, USA). Antibodies against AKT, pAKT (Ser 473), MMP-2, MMP-9, and inhibitor LY294002 were purchased from Cell Signaling Technology Inc. (Beverly, MA, USA).

**Figure 1:** The chemical structure of bufalin.

### Cell proliferation assay

HCCLM3 or HepG2 cells (1 × 10^4^) were plated into 96-well plates in triplicate and then treated with the indicated concentrations of bufalin. Cell proliferation was assessed after 48 h using CCK-8 (Dojindo, Tokyo, Japan) according to the manufacturer’s instructions. Results are expressed as the absorbance of each well at 450 nm (OD = 450).

### Wound healing assay

To determine cell motility, HCCLM3 and HepG2 cells were seeded separately into 24-well flat-bottomed plates and grown to 90% confluence. After aspirating the medium, the monolayer was scraped with a sterile micropipette tip to create a denuded zone with a constant width. The cells were then washed with phosphate-buffered saline (PBS) twice and exposed to the indicated concentrations of bufalin (0, 1, 10, or 100 nmol/L). The distances of wounds were monitored and photographed at 0, 24, and 48 h after treatment. Cell motility was calculated by the following formula: Cell motility = (distance at 24 or 48 h – distance at 0 h) / distance at 0 h.

### Transwell-migration/invasion assay

Cell migration was analyzed in a Transwell permeable support system (Corning Inc., Corning, NY, USA) containing 24-well transwell (unit 8 μm pore size polyvinylidene fluoride) filters. HCCLM3 and HepG2 were pretreated with 0, 1, 10, or 100 nmol/L bufalin for 48 h and then seeded into the upper insert at densities of 1 × 10^5^ cells/24-well for HCCLM3 and 5 × 10^4^ cells/24-well for HepG2 in serum-free DMEM. DMEM containing 10% FBS was added to the lower chamber as a chemoattractant. After culturing for 48 h, non-invading cells were removed from the upper surface by wiping with a cotton swab. The membrane was fixed with 4% formaldehyde for 15 min at room temperature. The invading cells were stained with Giemsa (Sigma, Munich, Germany) for 25 min, and their numbers in five fields of each triplicate filter were counted using an inverted microscope. The cell invasion assay was carried out similarly, except that 60 μl of 1:8 PBS-diluted Matrigel (BD Biosciences, Franklin Lakes, NJ, USA) was added to each well 6 h before cells were seeded onto the membrane.

### Cell adhesion assay

The 96-well flat-bottomed plates were precoated with 50 μl/well of 1:8 PBS-diluted Matrigel at 4°C overnight. After removing all coating solutions, the plates were blocked with 150 μl/well of 1% bovine serum albumin for 1 h at 37°C. Then HCCLM3 and HepG2 cells that had been treated with 0, 1, 10, or 100 nmol/L bufalin for 24 h were seeded into the Matrigel-coated wells at 1 × 10^5^ cells/well in triplicate and incubated for 4 h at 37°C in 5% CO_2_. After extensive washing, cells were fixed with 4% formaldehyde (100 μl/well) for 15 min and stained with a hematoxylin solution for 10 min. The average numbers of adhered cells in five fields were counted using an inverted microscope.

### Western blot analysis

The total and phosphorylated levels of AKT, GSK3β, and β-catenin and the protein levels of E-cadherin, MMP-9, and MMP-2 were evaluated by western blotting. Cells treated with bufalin were washed with ice-cold PBS and extracted in protein lysis buffer (Pierce, Rockford, IL, USA). Protein concentrations were determined with the BCA Protein Assay Kit (Beyotime, Shanghai, China). Protein samples of cell lysates were mixed with 5× sodium dodecyl sulfate (SDS) loading buffer (1:4), boiled for 5 min, and then separated on 8–10% SDS polyacrylamide gels. After electrophoresis, proteins were transferred onto polyvinylidene fluoride membranes, blocked in 5% nonfat dry milk in Phosphate Buffered Saline with Tween-20 (PBST) for 1 h, and incubated with corresponding rabbit monoclonal antibodies against pAKT (dilution 1:1000) and AKT (1:1000), pGSK3β (1:10000) and GSK3β (1:5000), pβ-catenin (1:500) and β-catenin (1:5000), E-cadherin (1:5000), MMP-2 (1:1000), MMP-9 (1:1000), and GAPDH (1:1000) overnight at 4°C. The membranes were washed three times with PBST and incubated for 1 h with a peroxidase conjugated secondary antibody. After washing again three times with PBST, blots were incubated with chemiluminescence substrate (ECL plus, Beyotime Inc., Shanghai, China), and digital images were acquired using a Chemi-Doc system employing Quantity One software (Bio-Rad Laboratories Inc., Hercules, CA, USA). Three independent blots were performed for each protein.

### Immunofluorescence

The expression levels of β-catenin and E-cadherin in bufalin-treated HCCLM3 and HepG2 cells were also evaluated by immunofluorescence. Cells were grown on glass cover slips to 60–80% confluence, and then fixed, permeabilized, and blocked. Cells were then incubated with primary rabbit monoclonal against E-cadherin and β-catenin overnight at 4°C. The next day, slides were washed and incubated with anti-rabbit fluorescein isothiocyanate-conjugated secondary antibody (Jackson, Lancaster, PA, USA). Cells were counterstained with 4′-6-diamidino-2-phenylindole to visualize cell nuclei and imaged by fluorescence microscopy (Olympus, Tokyo, Japan).

### Statistical analyses

Statistical analyses were performed with SPSS 17.0 for Windows (SPSS, Chicago, IL, USA). Quantitative variables are expressed as mean ± SD and were analyzed by analysis of variance. Results were considered statistically significant at *P* < 0.05.

## Results

### Inhibitory effects of bufalin on hepatoma cell proliferation

To explore the effects of bufalin on hepatoma cell proliferation, HCCLM3 and HepG2 cells were treated with bufalin at doses ranging from 0 to 100,000 nmol/L. Bufalin dramatically decreased the proliferation of the two tested cell lines in a dose-dependent manner, especially when exposed to more than 10 nmol/L (Figure 2). The inhibitory ratio of bufalin on cell proliferation was significantly increased from 21.4% ± 2.4% to 87.1% ± 0.7% in HCCLM3 cells and from 35% ± 5% to 88.6% ± 1.6% in HepG2 cells after a 48-h treatment. The data suggest that bufalin has robust suppressive effects on hepatoma cell proliferation.

**Figure 2:** **Inhibition curves of bufalin on hepatoma cell proliferation.** Proliferation of HCCLM3 and HepG2 cells was significantly inhibited by bufalin in a dose-dependent manner, especially when exposed to more than 10 nmol/L. All data represent the mean ± SD (n = 3).

### Effects of bufalin on hepatoma cell migration/invasion

To examine the effects of bufalin on cell migration, we performed wound healing and transwell-migration assays using the same two hepatoma cell lines. All wound healing images representing cell migration capabilities were taken at the same magnification and time after bufalin treatments. At 48 h, the wound was healed approximately 65.8% ± 4.8% in HCCLM3 and 84.0% ± 5% in HepG2. Bufalin significantly reduced cell motility in both HCCLM3 and HepG2 compared with the control (Figure 3). After treatment of HCCLM3 and HepG2 with bufalin at 100 nmol/L for 48 h, only 23.6% ± 4.6% and 41.6% ± 1.4% of cells had migrated, respectively. The migration assay using the transwell-migration system also demonstrated that bufalin (10 and 100 nmol/L) effectively inhibited cell migration of HCCLM3 and HepG2 (Figure 4). Furthermore, a transwell-invasion assay was used to determine the invasive activity of tumor cells across the basement membrane. Our results revealed that bufalin significantly decreased the invasive potential of HCCLM3 and HepG2 in a dose-dependent manner (Figure 5).

**Figure 3:** **Effects of bufalin on wound healing ability of hepatoma cells.** After scratches were made, HCCLM3 cells **(A**, **C)** and HepG2 cells **(B**, **D)** were allowed to proliferate for another 24 and 48 h in the absence or presence of different concentrations of bufalin. Columns represent the mean of three individual experiments performed in triplicate; error bars represent SD. *P < 0.05, **P < 0.01, vs. controls.

**Figure 4:** **Effects of bufalin on the migratory ability of hepatoma cells.** Cell migration of HCCLM3 **(A**, **C)** and HepG2 **(B**, **D)** after treatment with indicated concentrations of bufalin for 48 h. Columns represent the mean of three individual experiments performed in triplicate; error bars represent SD. **P < 0.01, vs. controls.

**Figure 5:** **Effects of bufalin on the invasive ability of hepatoma cells.** Cell invasion of HCCLM3 **(A**, **C)** and HepG2 **(B**, **D)** after treatment with indicated concentrations of bufalin for 48 h. Columns represent the mean of three individual experiments performed in triplicate; error bars represent SD.**P < 0.01, vs. controls.

### Effect of bufalin on hepatoma cell adhesion

To investigate the effect of bufalin on cell adhesion to the extracellular matrix, adhesion assays using HCCLM3 and HepG2 cells were performed in the presence or absence of bufalin. Pre-incubation of hepatoma cells with bufalin (10 and 100 nmol/L) markedly inhibited the adhesion of HCCLM3 and HepG2 (Figure 6).

**Figure 6:** **Effects of bufalin on the cell adhesion ability of hepatoma cells.** Adhesion of HCCLM3 **(A**, **C)** and HepG2 **(B**, **D)** cells to Matrigel were markedly inhibited by bufalin at doses of 10 nmol/L and 100 nmol/L as compared with control group cells. **P < 0.01, vs. controls.

### Effect of bufalin on the expression of AKT in hepatoma cells

The PI3K/AKT signaling pathway is one of the most important cellular pathways regulating HCC progression and affects cell proliferation, motility, and survival [12,13]. Therefore, we investigated whether bufalin was able to modulate the protein expression of AKT and pAKT (Ser 473) in human hepatoma cells by western blot analysis. At a dose of 100 nmol/L, bufalin significantly downregulated the expression of pAKT in both HCCLM3 and HepG2 cells without affecting the total protein levels of AKT (Figure 7). LY294002, a potent inhibitor of AKT, also reduced the levels of pAKT in both hepatoma cell lines. Furthermore, bufalin inhibited the expression of pAKT in HCCLM3 in a time-dependent manner. Our results clearly indicate that bufalin can significantly inhibit the activities of AKT in human hepatoma cells.

**Figure 7:** **Effects of bufalin on AKT and pAKT (Ser 473) expression in hepatoma cells. (A)** HCCLM3 and HepG2 cells were treated with bufalin (100 nmol/L) and LY294002 (10 mmol/L) for the indicated times. GAPDH was used as a loading control. **(B)** Quantitative analysis of expression of AKT and pAKT (Ser 473). Columns represent the mean of three individual experiments performed in triplicate; error bars represent SD; LY represent LY294002. **P < 0.01, vs. controls.

### Effects of bufalin on GSK3β and β-catenin expression and β-catenin nuclear translocation in hepatoma cells

To further examine the molecular actions of bufalin, we investigated the downstream molecules of the PI3K/AKT signaling pathway after bufalin treatment. Bufalin significantly suppressed the phosphorylation of GSK protein (Ser 9) and increased GSK3β protein activation (Figure 8A, C). Activation of GSK3β induces ubiquitin-dependent degradation of β-catenin, which acts as an important regulator of cell motility, invasion, and adhesion [15]. Therefore, we investigated the effects of bufalin on the downstream molecule levels in hepatoma cells. However, no pβ-catenin was detected in bufalin-treated cells (data not shown), and no obvious changes were found in the protein levels of β-catenin (Figure 8B, D). According to an immunofluorescence assay, bufalin suppressed the nuclear translocation of β-catenin both in HCCLM3 and HepG2 cells, especially in the latter (Figure 8E, F). In addition, our results demonstrated that treatment with LY294002 also suppressed the nuclear translocation of β-catenin in the two cell lines. These results confirm that bufalin inhibited Wnt signaling by decreasing the nuclear translocation of β-catenin.

**Figure 8:** **Effects of bufalin on GSK3β, β-catenin levels, and nuclear translocation of β-catenin.** Protein levels of pGSK3β **(A**, **C)** and β-catenin **(B**, **D)** were analyzed by western blotting in bufalin-treated (100 nmol/L) hepatoma cells. LY294002 (10 μmol/L) was included as a positive control. GAPDH was used as a loading control. Nuclear translocation of β-catenin in bufalin- and LY29400-treated hepatoma cells **(E**, **F)** was monitored by immunofluorescence assay. Columns represent the mean of three individual experiments performed in triplicate; error bars represent SD; LY represent LY294002. **P < 0.01, vs. controls.

### Effects of bufalin on E-cadherin, MMP2, and MMP9 expression in hepatoma cells

Nuclear localization of β-catenin promotes the expression of E-cadherin-mediated cell adhesion, sequentially endows tumor cells with migratory and invasion properties, and contributes to metastasis [15]. Therefore, we further investigated the downstream molecular actions of E-cadherin after the inhibitory nuclear translocation of β-catenin. First, E-cadherin protein expression was investigated by western blotting after treatment with bufalin for 48 h at a dose of 100 nmol/L. We found that bufalin significantly increased E-cadherin expression in HCCLM3 and HepG2 cells. These results were also confirmed by an immunofluorescence assay (Figure 9A–D). Overexpression of E-cadherin in highly invasive cells may reduce tumor cell invasiveness by decreasing MMP-9 and MMP-2 expression [16,17]. Therefore, the protein expression levels of MMP-2 and MMP-9 were investi-gated by western blotting after treatment with bufalin (100 nmol/L) or LY294002 (10 μmol/L). Indeed, bufalin significantly decreased MMP-9 expression in HCCLM3 and HepG2 cells and MMP-2 expression in HepG2 cells. These results suggest that bufalin can regulate the expression of MMP-9 and MMP-2 at the transcriptional level in hepatoma cells.

**Figure 9:** **Effects of bufalin on expression of E-cadherin, MMP-9, and MMP-2 in hepatoma cells.** The protein levels of E-cadherin **(A**, **B)** and MMP-9 and MMP-2 **(E**, **F)** were analyzed by western blotting in HCCLM3 and HepG2 cells after exposure to bufalin (100 nmol/L) and LY294002 (10 μmol/L). GAPDH was used as a loading control. Immunofluorescence assay showed expression of E-cadherin after exposure to bufalin and LY294002 in the two hepatoma cell lines **(C**, **D)**. Columns represent the mean of three individual experiments performed in triplicate; error bars represent SD; LY represent LY294002. *P < 0.05, *P < 0.01, vs. controls.

## Discussion

Although 90% of cancer deaths are caused by metastasis, the pathogenesis and mechanisms underlying this event remain poorly defined [18]. Recent studies suggested that the epithelial to mesenchymal transition initiates cancer cell dissemination, inducing non-cancer stem cells to enter into a cancer stem cell-like state [19], and promotes metastatic seeding accompanying the down regulation of E-cadherin [20,21]. The activation of the PI3K/AKT signaling pathway is emerging as a central feature of the epithelial to mesenchymal transition [14]. AKT, which is downstream of PI3K, has been shown to suppress transcription of the E-cadherin gene. Hyperactivated AKT decreases cell–cell connections by phosphorylating GSK3β (Ser 9), which is followed by ubiquitination and degradation, and the elimination of GSK3β permits β-catenin to accumulate and localize in the nucleus [11]. β-catenin is an essential molecule in the canonical Wnt signaling pathway. Its nuclear stabilization inhibits the expression of E-cadherin and promotes mesenchymal phenotype maintenance, migration, and invasion of carcinoma cells [15]. A current literature review shows the importance of cross-talk between the PI3K/AKT and β-catenin pathways as a therapeutic target in treatment of malignant tumors [22].

The traditional Chinese medicine Chansu, which is obtained from the skin and parotid venom glands of toads, has been used as a therapeutic reagent for several malignant tumors, including HCC, non-small cell lung cancer, and pancreatic cancer in China [7]. In a pilot study of treatment with Chansu extracts, 40% of advanced cancers (6/15) had prolonged disease stability or minor tumor shrinkage [7]. However, bufalin, the major digoxin-like active component of Chansu, exhibits a variety of biological activities, including cardiotonic, anesthetic, blood pressure stimulatory, respiratory, and anti-neoplastic effects [23]. These unwanted side-effects may prevent its use in cancer treatment. The potential use of cardiac glycoside-like compounds for the treatment of cancer, initially investigated 40 years ago, was abandoned because of the toxicity of these compounds. However, in 1999, a Scandinavian oncologist suggested that tumor cell apoptosis was induced by digoxins at a concentration without toxicity in humans [24]. Therefore, these agents might be useful for the treatment of cancer.

Activation of the PI3K/AKT signaling pathway contributes to cell proliferation, survival, motility, and angiogenesis, processes that are responsible for tumorigenesis, invasion, and metastasis [25]. For this reason, many pharmaceutical companies and academic laboratories are actively developing inhibitors targeting PI3K, AKT, and other important components in this pathway. Recently, lipid-soluble cardiac glycosides such as bufalin and oleandrin have been suggested as potent agents that might be useful as AKT inhibitors [26,27]. Because bufalin was reported to play an inhibitory role on AKT phosphorylation in gastric cancer cells [10], we hypothesized that a similar biological function may also exist in hepatoma cells. Our research here demonstrated that bufalin inhibited the phosphorylation of AKT, which in turn inhibited cell proliferation, migration, and invasion in the two hepatoma cell lines, and revealed that bufalin was able to suppress the phosphorylation of GSK3β (Ser 9) and increase the activated form of GSK3β. Although no obvious changes were found in the protein levels of β-catenin, the nuclear accumulation of β-catenin was markedly blocked in the two hepatoma cell lines. In turn, the reduced nuclear accumulation of β-catenin significantly increased the transcription of the transmembrane protein E-cadherin. In addition, bufalin was also able to decrease MMP-2 expression, especially in HepG2 cells, and MMP-9 in both cell lines. These results confirm the previous observations that overexpression of E-cadherin in human prostate cancer and mouse skin cancer reduced tumor cell invasiveness by decreasing MMP-2 and MMP-9 expression levels [16,17]. Therefore, upregulation of E-cadherin and a concomitant reduction in MMP-2/MMP-9 might negatively regulate cell proliferation, cell invasiveness, cell adhesion of HCCLM3 and HepG2. Similar results were observed in both of these hepatoma cell lines, which indicate the importance of AKT/GSK3β/β-catenin/E-cadherin signaling in HCC.

In brief, our results suggest that AKT is the main regulatory protein of the AKT/GSK3β/β-catenin/E-cadherin signaling pathway, which regulates the expression and phosphorylation of GSK3β and the nuclear translocation of β-catenin. β-Catenin functions as a negative regulation of the downstream molecule E-cadherin, which modifies the expression of downstream target proteins MMP2, MMP9.

This signaling pathway activation and protein regulation are related to hepatoma cell proliferation, migration, invasion, and adhesion. Thus, bufalin exhibits multiple anti-tumor effects on hepatoma cells because the mechanisms underlying bufalin action appears to mediate AKT/GSK3β/β-catenin/E-cadherin signaling and affect regulation of protein expression.

## Conclusion

In summary, our results suggest that bufalin exhibits multiple anti-tumor effects in hepatoma cells. The mechanisms underlying bufalin action appear to mediate the AKT/GSK3β/β-catenin/E-cadherin signaling pathway. Bufalin is a promising anti-HCC agent, and further studies should be performed in patients with HCC, especially those with advanced-stage disease.

## Competing interests

The authors declare that they have no competing interests.

## Authors’ contributions

YKY and WZW conceived the project. DZQ organized the study, analyzed the effects of bufalin on cell proliferation, migration, invasiveness and adhesion, and helped to prepare the manuscript. ZJZ modified the manuscript and repeated some experiments. ZJZ and DZQ performed the statistical and cell signaling pathway analyses. WZW and YKY contributed to the interpretation of the results and helped to write the manuscript. All the authors read and approved the final manuscript.

## Pre-publication history

The pre-publication history for this paper can be accessed here:

http://www.biomedcentral.com/1472-6882/13/185/prepub
